RETRACTED

# A Study of Athlete Pose Estimation Techniques in Sports Game Videos Combining Multiresidual Module Convolutional Neural Networks

**DOI:** 10.1155/2021/4367875

**Published:** 2021-12-28

**Authors:** Rui Liu

**Affiliations:** Department of Physical Education, Lvliang University, Shanxi Lvliang 033001, China

## Abstract

In this paper, we propose a multiresidual module convolutional neural network-based method for athlete pose estimation in sports game videos. The network firstly designs an improved residual module based on the traditional residual module. Firstly, a large perceptual field residual module is designed to learn the correlation between the athlete components in the sports game video within a large perceptual field. A multiscale residual module is designed in the paper to better solve the inaccuracy of the pose estimation due to the problem of scale change of the athlete components in the sports game video. Secondly, these three residual modules are used as the building blocks of the convolutional neural network. When the resolution is high, the large perceptual field residual module and the multiscale residual module are used to capture information in a larger range as well as at each scale, and when the resolution is low, only the improved residual module is used. Finally, four multiresidual module convolutional neural networks are used to form the final multiresidual module stacked convolutional neural network. The neural network model proposed in this paper achieves high accuracy of 89.5% and 88.2% on the upper arm and lower arm, respectively, so the method in this paper reduces the influence of occlusion on the athlete's posture estimation to a certain extent. Through the experiments, it can be seen that the proposed multiresidual module stacked convolutional neural network-based method for athlete pose estimation in sports game videos further improves the accuracy of athlete pose estimation in sports game videos.

## 1. Introduction

There is a huge market demand for the analysis and understanding of sports game videos. It can improve the shooting method of sports game video so that viewers can enjoy clearer and more professional sports game video images, it can target the performance on the sports field so that viewers can hear more wonderful commentary, and it can also provide standard teaching cases for the majority of sports fans [1]. In addition, statistics of various data of athletes in sports game videos can not only help athletes improve their technical level but also adjust tactical deployment for the whole team in a targeted way. For example, in large sports such as basketball and soccer, statistics of players' running distance and trajectory and analysis of athletes' human posture in swimming and diving can help coaches and athletes improve the strength of the team to a certain extent [2]. The demand for analysis and understanding of sports game videos is increasing, but with the explosive growth in the number of sports game videos, it has been difficult for the traditional manual annotation-based sports game video analysis methods to meet this expanding demand due to their high cost and many limitations [3]. The target detection technique can detect the position of athletes, the target tracking technique can count the athletes' motion trajectory, and the athlete pose estimation can identify the athletes' pose. Target detection and athlete pose estimation for sports game videos are the basis for the analysis and understanding of sports game videos. Existing techniques for target detection and athlete pose estimation have achieved good performance on generic picture-based scene detection tasks, but there are few algorithms and data dedicated to targeting detection for sports game video scenes. For a new data domain, it is common practice to annotate this data and then train the target detection algorithm with the new data to obtain a detection model [4].

RETRACTED

With the continuous development of the Internet, a large amount of sports game video data emerges every day, which brings us rich information resources but also poses a huge challenge to retrieve the data we need. Although computer hardware devices are constantly updated, it is still a huge challenge to face the computational burden brought by the large-scale sports game video retrieval task. Most previous sports game video retrieval is based on keyword retrieval, while content-based sports game video retrieval is a more popular research topic, which can well understand various parameters, features, and other information of human action in sports game video, match the corresponding action patterns, and then retrieve them in the network data [5]. Athlete pose estimation techniques can better help computers understand human movements in sports game videos and combine relevant joint and pose information to enable computers to quickly retrieve the desired sports game videos. Within the field of practical athlete pose estimation research, athlete pose estimation is divided into two-dimensional based pose estimation and three-dimensional based pose estimation according to the different spatial dimensions of the research; according to the number of people, athlete pose estimation is divided into single-person pose estimation and multiplayer pose estimation; this paper only discusses the research in the direction of single-person pose estimation based on two-dimensional static images, and effective athlete pose estimation must not only detect human parts or joints from the image to be measured but also correctly locate the specific positions of these parts or joints; in addition, it must be able to handle large limb changes, changes in clothing and lighting conditions, and severe human occlusion problems [6]. Therefore, athlete pose estimation is a popular research topic in the field of computer vision that is both valuable and extremely challenging to study [7].

RETRACTED

This paper mainly studies the detection of athletes and human pose estimation in sports videos. Starting from image-based target detection and human pose estimation algorithms, combined with the characteristics of sports videos, the target detection and human pose estimation models trained based on general data sets are migrated. In the field of sports video, it aims to reduce the cost of training and labeling for sports video-oriented athlete detection and pose estimation tasks and at the same time improve the performance of athlete detection and human pose estimation in sports videos. The first section of this paper is an introduction, which introduces the current research status in the field of athlete pose estimation and the main challenges encountered in the field of human action recognition and introduces many research implications of athlete pose estimation and the research framework of this paper. The second section is a study of related work; firstly, it gives a detailed introduction to the research status of convolutional neural network for athlete pose estimation in sports game video and describes the key directions of this paper.  Section 3 proposes a multiresidual module convolutional neural network-based athlete pose estimation method, which uses three different residual modules to effectively capture the image feature information as well as visual information of the image at each scale and then predict the joint coordinates more accurately.  Section 4 is the analysis of experimental results, where we describe in detail the design and operation of the whole experiment and analyze some problems encountered in experimenting on a public dataset. The relevant experimental settings and performance metrics, as well as the experimental results, are analyzed and discussed. The experimental results show that our model can more comprehensively and accurately locate some key points that are difficult to detect in 2D multiperson pose estimation and has better robustness, laying the foundation for subsequent human behavior recognition and understanding.  Section 5 is the conclusion, which summarizes the research content of the whole paper and provides a description and outlook for future research.

RETRACTED

## 2. Related Work

Athlete pose estimation has applications in many computer vision tasks, such as motion recognition, video surveillance of sports competitions, and human trajectory tracking. Given a sports game video or a sequence of pictures, the task of athlete pose estimation is to estimate the positions of the joints of human instances in the scene [8]. The deep learning-based athlete pose estimation algorithm views human pose detection as a key point regression problem and is trained with a large amount of data with joint point class and position annotations to finally obtain a model that can predict the position and class of human joint points. Bazarian et al. designed an hourglass-like network structure for pose detection and added a supervisory signal in the middle of the network to improve the pose detection accuracy [9]. Mundt et al. introduced a feature pyramid to perform nodal regression at multiple scales to obtain more accurate nodal positions [10]. The single-person pose estimation task uses only one human pose detection with a simple image background and less interference, and the existing single-person pose estimation algorithms have achieved good performance, reaching over 93% accuracy on the single-person pose estimation dataset MPII [11]. However, in practical situations, most of the images have multiple human bodies in them, when the single-person pose estimation algorithm is no longer applicable.

For the technique of multiresidual module convolutional neural network for pose estimation of athletes in sports video, the main process of the algorithm is as follows: the feature extraction network extracts the candidate's joints, and the extracted joints are grouped using an integer linear programming formulation, which is a bottom-up algorithm. Wang used ResNe network to replace the main network for candidate's joints. They also pointed out the coupling constraints for image conditions, reduced the number of candidate nodes, optimized the Deep Cut algorithm, and used the Deeper Cut algorithm for pose estimation [12]. Yuan et al. proposed the top-down Mask RCNN algorithm, which has achieved good results in target detection experiments [13]. The algorithm is also applicable to the field of athlete pose estimation. With the rapid development of deep learning and convolutional network technology, the accuracy of athlete pose estimation for relatively simple and standard normal pose has been significantly improved, but for some special complex pose or multiperson pose in masking situations, existing methods still have problems such as inaccurate positioning of joints and incorrect connection of associated joints [14]. Researching methods that can solve both simple athlete pose estimation and complex athlete pose estimation problems is an urgent problem at present; in particular, the correct estimation of the complex pose has more important application value in practice [15, 16].

RETRACTED

In general, the existing athlete pose estimation algorithms have achieved good performance, but there are still some problems in some specific scenarios, such as top-down multiperson pose estimation algorithms when multiple people are gathered and obscured which will produce missed and false detections [17, 18]. At the same time the existing athlete pose estimation algorithm is designed based on the generic human body, which will detect all the human poses in the figure; when some specific areas of detection often only need the pose of a specific human body, the existing algorithm cannot further differentiate the human pose. In practice, many domains wait for only the pose of a specific individual, such as the pose of an athlete in a sports video and the pose of an actor on a stage. The existing algorithms are more concerned with the accuracy of detecting multiple human poses, and there are few studies on the detection of specific human poses [19, 20]. Most of the existing datasets are generic datasets, which will contain many common scenarios of life, and the models trained based on these datasets already have the potential to detect these domain-specific targets, only that there is no more detailed distinction in the detection results. For example, detecting athletes in a sports game video can be seen as the detection of people in a sports scene, except that the generic detector cannot identify the athletes in the detection results [21]. The athlete pose estimation method based on the multiresidual module convolutional neural network proves its significant advantages over traditional methods and can obtain higher pose estimation results. However, how to design a dedicated network structure with higher accuracy and robustness for the athlete's pose estimation problem has become an emerging research direction [22]. In this paper, we will investigate the human detection model trained based on the generic dataset and migrate it efficiently to the sports game video domain to complete the detection and pose estimation of athletes in sports game videos [23].

## 3. Research on Athlete Pose Estimation Technique in Sports Game Video based on a Convolutional Neural Network with Multiple Residual Modules

### 3.1. Multiresidual Module Convolutional Neural Network Model Construction

The design and use of residual learning improve the performance of the network while also improving the accuracy of the athlete's pose estimation task. It mainly uses the unit mapping in the residual module to simplify the deep network parameters, allowing us to train very deep neural networks, but the unit mapping is also the source of the drawback of residual learning: the unit mapping keeps increasing the variation of the response as the network goes further, thus increasing the optimization difficulty [24]. In convolutional neural networks, the impact of increasing response will be more obvious because the building blocks of hourglass subnetworks are dominated by residual modules, and multiple hourglass subnetworks cascade to form convolutional neural networks. It can be imagined that the main module used in the whole convolutional neural network is the residual module, and thus the response in the network has a greater impact during the training of deep networks like convolutional neural networks, which leads to network parameters being difficult to optimize, which eventually affects the prediction accuracy [25].

RETRACTED

Among other tasks in computer vision, dropout is a simple and effective regularization technique in neural networks and deep learning models, which can effectively prevent overfitting while improving the generalization ability of the model [26, 27]. Since this section uses a fully convolutional network, and there is a strong spatial correlation between each joint point feature and part feature of the human body on the training image, the feature map activation also has a strong. In this case, by introducing spatial dropout, it can help the network to learn the correlation between adjacent pixels on the feature map, and it can well prevent overfitting during the training process of the network and optimize the performance of the network. This article collects and organizes sports game videos and selects 10 complete sports games as the original video data. The total video duration reaches 2088 minutes. Because there will be many ads, interstitials, and pauses in the complete video and the length of the video will cause too much processing time, this article segmented the complete video. Using video editing tools that do not affect the image quality, we will intercept every complete game video. Each game will intercept 20 segments, each time is 10–20 seconds, and a total of 200 videos with a total duration of 678 seconds will be obtained. Then these video clips are divided into frames, and the size is set to 1100_ _×_ _700 pixels, and a total of 17,850 pictures are obtained.

The use of two separate 3*∗*3 filters instead of one 5*∗*5 filter allows for better learning of spatial context information, and therefore no convolutional layer with a convolutional kernel size larger than 3*∗*3 is used in all residual modules, thus reducing the total number of parameters in the network. Although the proposed improved residual module improves the model performance, the effective perceptual field of the improved residual module is smaller due to the smaller size of the convolutional kernel in this residual module, and the large perceptual field residual module is designed based on the improved residual module to better learn the correlation between human nodes. Deep residual learning has made significant breakthroughs in image recognition and classification tasks by using residual modules, which can be expressed as

(1) $$\begin{array}{c} M_{i+1}=\alpha *H\left(M_{i}\right)+\beta *G\left(M_{i},W_{i}^{g}\right), \end{array}$$

where *M*_i_ and *M*_*i* + 1_ are the input and output of the *i*-th residual module, respectively, and *G* is the convolution of the stack, normalized, and relu, where *H*(*M*_*i*_) = *M*_*i*_ is the unit mapping. The expression of the designed large-feeling wild residual module is shown in the following equation:

(2) $$\begin{array}{c} M_{i+1}=\alpha *H\left(M_{i}\right)+\beta *G\left(M_{i},W_{i}^{g}\right)+\gamma *P\left(M_{i},W_{i}^{p}\right). \end{array}$$

The improved residual module can avoid the effect of unit mapping in the traditional residual module, and the large perceptual field residual module expands the perceptual field of the network output layer, but these two residual modules cannot essentially solve the problem of inaccurate node localization due to the change of human scale in the image. This section proposes a multiscale residual module based on the large perceptual field residual module; as the name implies, the multiscale residual module can learn the feature information of the image at multiple scales, and it mainly consists of convolution layer, normalization layer, activation layer, pooling layer, upsampling layer, and spatial dropout layer, as shown in Figure 1.

RETRACTED

The expression of the module is shown in the following equation:

(3) $$\begin{array}{c} M_{i+1}=\alpha *H\left(M_{i}\right)+\beta *G\left(M_{i},W_{i}^{g}\right)+\gamma *P\left(M_{i},W_{i}^{p}\right)+\lambda *Q\left(M_{i},W_{i}^{q}\right). \end{array}$$

In the sports competition athlete posture evaluation data set, 17 human body joint points need to be predicted, namely, left ear, right ear, left eye, right eye, nose, left shoulder, right shoulder, left elbow, right elbow, left wrist, right wrist, left hip, right hip, left knee, right knee, left ankle, and right ankle; this article uses the same method to label these 17 joint points. In this paper, 100 pictures are randomly selected from the pictures with borders to mark the joint points of the athletes, a total of 773 personal postures.

### 3.2. Optimization of Athlete Pose Estimation Algorithm

Recognition of athletes, that is, distinguishing between athletes and nonathletes, is essentially a matter of classifying candidate frames based on their features. Define a feature vector *q* to represent athletes, and let the candidate box features of athletes be close to *q* and the candidate box features of nonathletes be far from *q*. This allows setting a threshold to distinguish athletes from nonathletes. From the candidate frame selection and feature extraction module, the 2048-dimensional depth feature corresponding to each detection frame can be obtained, which can be used to distinguish different detection frames but cannot distinguish athletes from nonmobilizers, so a linear transformation of these features is needed, and this linear transformation module transforms the 2048-dimensional candidate frame features into new 512-dimensional features. A 512-dimensional feature vector *q* is initialized to represent athletes, and by continuously optimizing the parameters of this linear transformation module, the new features of athlete candidate frames can be made more similar to *q* and the new features of nonathlete candidate frames can be made less similar to *q*. The formula of this linear transformation module is as follows:

(4) $$\begin{array}{c} T=f\left(w*t_{2048}\right). \end{array}$$

In equation (4), *t*_2048_ denotes the original 2048-dimensional feature of the candidate frame, *T* denotes the new 512-dimensional feature after linear transformation, *f* is the activation function of the linear transformation module, and *w* is the weight parameter of the linear transformation module. Suppose *M* denotes the athlete and *N* denotes the picture containing the athlete; then the positive packet similarity can be expressed as *F*(*M*, *N*) and *K* denotes the picture without the athlete; then the negative packet similarity can be expressed as *F*(*M*, *K*). The similarity between the pictures containing athletes and the category of athletes is greater than that of pictures without athletes, *F*(*M*, *N*) > *F*(*M*, *K*). Thus the loss function of this multiexample learning model is defined as

(5) $$\begin{array}{c} \text{Loss}=\max\left(F\left(M,N\right)-F\left(M,K\right)+\beta ,0,\min\left(F\left(N\right),F\left(K\right)\right)\right). \end{array}$$

In equation (5), *β* denotes the similarity differentiation interval and max is the function of taking the maximum value. In the convolutional neural network, the accurate localization of key points of the human skeleton has a high requirement on the size of the effective receptive field area. The expression of the receptive field is shown in the following equation:

(6) $$\begin{array}{c} f\left(Ki+1\right)=F\left(i\right)*\left(f\left(K_{i}\right)-1\right)+N_{i}. \end{array}$$

In equation (6), *f*(*K*_*i*_) is the receptive field of the *i*-th convolutional layer, *f*(*K*_*i* + 1_) is the receptive field on the *i* + 1-th layer, *F* is the step size of the convolution, and *N* is the current layer convolutional kernel size. In the human visual system, humans focus their eyes on the object they want to focus on while ignoring some irrelevant information. The attention mechanism is a way to present the key information more directly and completely. By introducing the attention mechanism into the athlete's pose estimation task, the key information in the image, the human body region, can be focused on, while the background interference is filtered out to improve the model detection accuracy. The mathematical principle of the attention mechanism is as follows:

(7) $$\begin{array}{c} G\left(a,b,c\right)=\sum_{i=1}^{N}\frac{\sum_{j=1}^{N}\ln\left(F\left(a_{j},c\right)\right)}{\ln\left(F\left(a_{i},c\right)\right)}. \end{array}$$

In equation (7), *a*, *b* denote key-value pairs, *c* is the query vector, and *F* is the attention score. The attention mechanism starts by generating the overall features as in the following equation:

(8) $$\begin{array}{c} \beta =f\left(c+w⊕a\right)+g\left(c+w⊙b\right). \end{array}$$

In equation (8), *β* is the overall information feature, *f* is the nonlinear activation function, and ⊕ and ⊙ are the convolution operation. After softening the activation function of the mask branch, the approximate mask range of the human body region can be obtained, as in equation (9), where *F* is the human body region, and *β* is the attentional feature map:

(9) $$\begin{array}{c} \beta \left(x,y\right)=\sum_{i=1}^{N}\frac{e\left(x,y\right)}{F^{e\left(x_{i},y_{i}\right)}}. \end{array}$$

RETRACTED

### 3.3. Athlete Pose Estimation System Design Implementation

In the prototype system of athlete pose estimation, firstly, the sports game video dataset is input to the system as the data source, then the desired athlete pose estimation model is selected to detect the key points for each second appearing in the sports game video, and finally, the detected results are output. The prediction result of the prototype system consists of three parts: the first part is the detection frame for the target person, along with the person class labeled in the upper left corner; the second part is the line of human key points, which constitutes the human pose; and the third part is the detection time labeled in the upper left corner of the detection frame. The prototype system can get the prediction result of the current second by pausing the sports video, and the detection time of each second is relatively fixed. However, when the human body is occluded, then there is no great impact on the prediction of the detection frame, but it will affect the detection of key points in the occluded part, making the connection between the joints incomplete. For different times in the sports game video, the human body key points can be detected. Meanwhile, the prototype system uses sports game video editing techniques to stitch the prediction results into separate sports game videos according to different target characters appearing in the sports game videos. The software architecture of the human posture evaluation system is shown in Figure 2.

The design of the hardware parameters focuses on the camera placement angle and the parameters of the camera itself. The software interface part of the design focuses on the camera interface layer. Since many camera drivers are developed independently, resulting in inconsistent drivers used by the cameras, the human posture evaluation uses a camera interface layer designed to be compatible with the drivers.

In the training process, the input layer (input) of this optimization model has two parts: one part is the input image matrix, the images are transformed from dimensions (height, width, and number of channels) to (number of images, height, width, and number of channels) by cutting, rotating, and masking operations; the other part is the mask, which provides the ROI region of the human body in the training set when making the dataset. Each frame in the dataset already contains the grayscale image of human limbs and the grayscale image of human skeletal points in the preset image. The dataset is used first during training and the model weight parameters are saved at the end of training. This is the first training to ensure the accuracy of the optimization model for estimating the generic human pose by training on the dataset. Subsequent training does not use the initialized weights but reads the weight parameters from the first training and uses the collected athlete images for training based on this dataset to ensure the accuracy of the optimization model for estimating the human posture of the athlete.

## 4. Results and Analysis

### 4.1. Multiresidual Module Convolutional Neural Network Model Analysis

The larger the PCKh (in MPII, head length is used as a normalized reference) value is, the higher the recognition accuracy is. The recognition accuracy of the model in this paper is higher than that of Deepercut, SHN, and CPM with LSP as the training set. The recognition accuracy in the head, shoulder, elbow, wrist, and hip parts is the same as that of CPM with MPII as the training set and slightly lower than that of the best HRnet model, but the recognition accuracy in the knee and ankle parts is higher. In terms of model complexity, HRnet >CPM > Deepercut > SHN; therefore, it can be concluded that this model has a greater advantage in solving the repetitive counting problem and the inverse order problem of joint points in the field of athlete pose estimation and can better introduce the physiological feature information to improve the recognition effect of athlete pose estimation. The overall athlete pose estimation results are better in both subjective visual and objective indicators. In addition, the recognition accuracy of the CPM algorithm with MPII as the training set is higher than that of the CPM model with LSP as the training set, which proves that the more the data types are included in the data set, the better the estimation results are (Figure 3).

RETRACTED

To illustrate the experimental rigor and to demonstrate the robustness of the model, we further tested our model on the test set test-dev2020 of the dataset. In Figure 4, we show the test results of our network model on the test set test-dev2020. The residual module model still outperforms Simple Baseline (ResNet50) on test-dev2020, with AP of 70.7, an improvement of 0.7; APL of 76.7, an improvement of 0.9; AR of 76.4, an improvement of 0.8; ours+  model on test-dev2020. The results of ours + model on test-dev2020 have also been further improved. Compared with Simple Baseline (ResNet50), the AP of the large perceptual field residual module model is 71.1, an improvement of 1.1; AP50 is 91.0, an improvement of 0.1; APL is 76.9, an improvement of 1.1; and AR is 76.6, an improvement of 1.0. The improved large perceptual field residual module model on test-dev2020 is also improved. The improved large perceptual field residual module model on test-dev2020 also improved again. Compared with Simple Baseline, the AP of the improved large perceptual field residual module model is 71.7, an improvement of 1.7; AP50 is 91.2, an improvement of 0.3; APL is 77.5, an improvement of 0.9; and AR is 77.3.

Based on the above results, we can see that our joint local and global structure and jump connection module can effectively improve the performance of the model on the 2D multiplayer pose estimation task with some robustness. Overall, the improved large perceptual field residual module model has improved all metrics on the test-dev2020 dataset, where the improvement of AR indicates that ours++ model is indeed able to detect some key points that are not detected, while the improvement of AP, AP50, and AP75 indicates that the improved large perceptual field residual module model can have a more accurate localization. In addition, the improved large perceptual field residual module models APM and APL are also improved, but the test results of APM for medium-sized targets are still smaller than those of APL for large-sized targets, which again supports the importance of local details in the 2D multiperson pose estimation task.

RETRACTED

### 4.2. Performance Analysis of the Athlete Pose Estimation Algorithm

In the experimental verification on the MPII data set, the method in this section is compared with the Open-Pose, Hourglass, and MSPN methods, and the results are shown in Table 1. It can be seen from Table 1 that the human posture estimation model IPR-DDHPE optimized by integral posture regression can significantly improve its prediction accuracy at key points such as head and shoulder. Its average accuracy mAP can reach 94.6%, which is better than that shown in Table 1. Other models are listed.

The LSP dataset is jointly trained with the MPII dataset in the experiments, and the performance is tested on the LSP test set, and the final results of the comparison experiments are given under both PCK and PCP criteria, and the results of other athlete pose estimation methods are taken from the corresponding references. The results of the comparative experimental data under the PCK criterion are given in Figures 5(a).  Figure 5(b) gives the experimental data results for the LSP test set under the PCP criterion.

In this section, the experiments compare MRSH with athlete pose estimation methods commonly used in recent years. The experiments use the MPII dataset for model training, and since the test set of the MPII dataset is not publicly available, the results of the tests are submitted to MPU, which provides feedback on the final prediction results. The final results of the comparison experiments under the PCKh criterion are given, and the data results of other athlete pose estimation methods are also provided by MPU. The results of the comparison experimental data under the PCKh criterion are given in Figure 6.

According to the data results in Figures 5 and 6, it can be seen that the MRSH method proposed in this section is competitive compared with advanced athlete pose estimation methods and achieves high prediction accuracy in both the LSP dataset and MPII dataset, where the PCP criterion is a measure of the accuracy of the body part estimation, and the upper arm and lower arm are most affected by occlusion in the LSP dataset, as can be seen from the data in Figure 5. The MRSH proposed in this paper achieves high accuracy of 89.0% and 82.5% in the upper arm and lower arm, respectively, so the method in this section reduces the effect of occlusion on the estimation of the athlete's posture to some extent. In addition, according to the data results in Figure 5, the proposed MRSH method based on the traditional hourglass network for the problem of the influence of the variation of the scale of human parts on the pose estimation accuracy has further improved the accuracy of the athlete pose estimation compared with the SDCNN method proposed in Section 3. Therefore, the MRSH proposed in this section contributes to the improvement of the test accuracy of the athlete's pose estimation, and it achieves such a good result under the limited experimental equipment because the MRSH is designed considering the influence of the part size and the advantage of the large perceptual field for the reasoning of the obscured human joints. Therefore, MRSH can fully learn the feature information at different scales during training and learn the correlation between joints in a large enough receptive field, which greatly improves the accuracy of athlete's pose estimation.

RETRACTED

### 4.3. Application Analysis of Athlete Pose Estimation System

For the human pose evaluation module using 6 sports videos, the number of frames in each sports video where the pose should be detected is called the “number of frames to be measured,” and the number of frames in each sports video where the pose is detected is called the “number of frames measured.” The comparison of the data is shown in Figure 7.

To evaluate the effect of the step modules in the SDCNN designed in this paper on the performance of human pose estimation, this section is conducted separately on the FLIC dataset using different numbers of step modules under the same conditions of other experimental settings.  Figure 8 gives the experimental data results of the SDCNN trained model composed of different numbers of step modules under two evaluation criteria, PCP and PCK, with a PCK threshold of 0.2 and PCP threshold of 0.5, for all experiments in this paper.

From the experimental results, we can see that when the number of step modules gradually increases, the performance of the corresponding SDCNN trained model on the human pose estimation task also keeps improving, and when the number of step modules increases to 4, the trained model tests out with higher accuracy, and after a large number of experiments of increasing the number of step modules, we find that when the number of step modules continues to increase, the test results in there show no significant improvement in the accuracy values. The final number of ladder modules for the best network used on the FLIC data set is 4, while the number of ladder modules for the best network used on the LSP data set is 5.

RETRACTED

## 5. Conclusion

This paper proposes a multiresidual module convolutional neural network-based athlete pose estimation method, which uses three different residuals compared with the advanced athlete pose estimation methods. In addition, the use of intermediate supervision also avoids the problem of gradient disappearance in the network training process. The experimental results show that the accuracy of the proposed MRSH for testing human parts and joints is improved. The method is based on the detection frame of the athlete first preprocessing the image to remove the background of nonathletes and then using the bottom-up pose detection idea to complete the pose estimation of athletes in sports competition videos, which improves the detection speed while reducing the missed detection. In this paper, we have explored the athlete detection and pose estimation algorithms for sports game videos, and we have made some progress in improving model reusability and reducing labeling and training costs. The method in this paper detects every frame of sports game video, and the detection results are still somewhat different in different sports game video frames, even though the two frames are adjacent and the contents are similar. When the results are drawn for the sports game video frames, the detection frame of the same athlete will be jittered. To improve the visual effect, the introduction of a sports game video tracking strategy for the detection frames can be considered.

## Figures and Tables

**Figure 1:** Schematic diagram of MSRM.

**Figure 2:** The software architecture of the body attitude evaluation system.

**Figure 3:** Model run time.

**Figure 4:** Test results on test-dev2020.

**Figure 5:** Comparison results on the LSP dataset. (a) Comparative experimental data under the PCK standard. (b) Comparative experimental data under the PCP standard.

**Figure 6:** Comparison results of PCKh on MPII dataset.

**Figure 7:** The measured frame rate of sports video.

**Figure 8:** Attitude estimation results.

**Table 1:** Experimental results of the model on the MPII dataset.

Algorithm	Head	Shoulder	Elbow	Wrist	Hip	Knee	Ankle	mAP
Open-pose	91.32	87.63	77.80	66.84	75.41	68.99	61.74	75.70
Hourglass	98.42	96.32	91.26	87.16	90.12	87.41	83.63	90.91
MSPN	98.64	97.18	93.25	89.27	92.09	90.16	85.54	92.61
Research algorithm	99.24	98.31	94.69	90.11	94.50	93.29	86.42	94.69

## Data Availability

The data used to support the findings of this study are available from the corresponding author upon request.
